# AMPA Receptor Trafficking in Natural and Pathological Aging

**DOI:** 10.3389/fnmol.2017.00446

**Published:** 2018-01-09

**Authors:** Sandra Jurado

**Affiliations:** Instituto de Neurociencias CSIC-UMH, San Juan de Alicante, Spain

**Keywords:** AMPAR receptors, aging, neurodegenerative diseases, Alzheimer’s disease, synaptic transmission

## Abstract

α-amino-3-hydroxy-5-methyl-4-isoxazolepropionic acid receptors (AMPARs) enable most excitatory transmission in the brain and are crucial for mediating basal synaptic strength and plasticity. Because of the importance of their function, AMPAR dynamics, activity and subunit composition undergo a tight regulation which begins as early as prenatal development and continues through adulthood. Accumulating evidence suggests that the precise regulatory mechanisms involved in orchestrating AMPAR trafficking are challenged in the aging brain. In turn dysregulation of AMPARs can be linked to most neurological and neurodegenerative disorders. Understanding the mechanisms that govern AMPAR signaling during natural and pathological cognitive decline will guide the efforts to develop most effective ways to tackle neurodegenerative diseases which are one of the primary burdens afflicting an increasingly aging population. In this review, I provide a brief overview of the molecular mechanisms involved in AMPAR trafficking highlighting what is currently known about how these processes change with age and disease. As a particularly well-studied example of AMPAR dysfunction in pathological aging I focus in Alzheimer’s disease (AD) with special emphasis in how the production of neurofibrillary tangles (NFTs) and amyloid-β plaques may contribute to disruption in AMPAR function.

## Introduction

The α-amino-3-hydroxy-5-methyl-4-isoxazolepropionic acid receptors (AMPARs) are glutamate-gated channels that mediate most fast excitatory transmission in the central nervous system (CNS). Because of their crucial role in regulating brain function, AMPARs are under tight regulatory processes that control their biosynthesis, membrane trafficking, degradation and various post-translational modifications (Anggono and Huganir, 2012; Lu and Roche, 2012). Arguably, one of the most important functions of AMPAR dynamics might be to underlie several forms of synaptic plasticity which has been proposed to act as a subcellular correlate of learning and memory (recently reviewed in Huganir and Nicoll, 2013; Nicoll, 2017). Significant advances over the last decades have contributed to our understanding of the processes involved in AMPAR dynamics at synapses, nonetheless how these mechanisms regulate normal synaptic transmission and plasticity and how they go awry during natural aging and neurodegeneration remain unknown.

Elucidating the underlying mechanisms of brain function and decline is especially relevant in today’s society since an increasingly aged population faces higher risks of developing neurodegenerative diseases such as Alzheimer’s disease (AD). In the U.S. alone, AD affects more than 5 million people with an annual cost of over 200 billion^1^. Over the last two decades researchers have exposed subtle differences in synaptic structure and function at early stages of AD in accord with the notion that subcellular reorganization precedes actual neuronal loss (Coleman and Flood, 1987; Brown et al., 1998; Scheff et al., 2006; Shankar et al., 2007). Consistently, one of the earliest biological manifestations of AD dementia is reduced synaptic AMPARs and synaptic plasticity impairments (Walsh et al., 2002; Shankar et al., 2008; Li et al., 2009; reviewed in Burke and Barnes, 2006; Guntupalli et al., 2016).

At the molecular level, AD is characterized by the presence of two pathological metabolites: plaques formed by oligomeric clusters of amyloid-β (Aβ) and neurofibrillar tau tangles (NFTs). Aβ is a secreted proteolytic derivative of the amyloid precursor protein (APP) which has been linked to early deficits in AD pathogenesis (Lambert et al., 1998; Lesné et al., 2006). NFTs are aggregates of hyperphosphorylated tau, a protein essential for microtubule assembly (Cleveland et al., 1977; Harada et al., 1994) whose aberrant conformation has been proposed to induce neurotoxicity. Together with Aβ, NFTs is considered a hallmark of AD but tangles can be found in different neurodegenerative diseases known with the general name of tauopathies. A large body of work has deepened our knowledge of how these pathological metabolites alter AMPAR dynamics to undermine synaptic function. Furthermore there has been a growing appreciation that Aβ and NFTs may synergistically act to disrupt synaptic AMPARs. Nonetheless, the mechanisms employed by Aβ and NFTs to hijack synaptic transmission and plasticity are only partly understood. In this review, I provide a brief overview of the current models of AMPAR trafficking to then focus on how these processes may be altered by both Aβ and NFTs.

## Mechanisms of AMPAR Trafficking: A Brief Overview

Given their critical role, the mechanisms underlying AMPAR dynamics during baseline transmission and plastic events have been the focus of extensive study over the last decades. Particularly AMPAR trafficking during synaptic plasticity has drawn the most attention. The term synaptic plasticity refers to neurons’ ability to adapt the strength of synaptic responses as a consequence of changes in neuronal activity. Among several different types of plasticity, the best known is a bidirectional form of Hebbian plasticity that requires the activation of N-methyl-D-aspartate receptors (NMDARs) that triggers AMPAR mobilization. A prominent example of this form of plasticity is long-term potentiation (LTP). LTP is elicited in response to high frequency stimulation for brief periods of time (in the order of seconds) sufficient to activate NMDARs initiating a calcium-dependent mechanism that recruits synaptic AMPARs thereby increasing synaptic efficacy. Conversely, low frequency stimulation for several minutes leads to the removal of synaptic AMPARs to produce a long-sustained decrease in synaptic strength known as long-term depression (LTD). Both forms of NMDAR-dependent plasticity have been proposed to underlie important functions like information processing, learning and memory (reviewed in Huganir and Nicoll, 2013; Nicoll, 2017). In addition, synaptic AMPARs may be passively replenished by constitutive trafficking mechanisms (reviewed in Shepherd and Huganir, 2007; Henley et al., 2011). Here, I briefly introduce some of the most important findings regarding constitutive and regulated AMPAR trafficking to later discuss how these processes may be altered during AD.

### AMPAR Subunits and Synaptic Plasticity

AMPARs are tetrameric assemblies of two dimers of four subunits (GluA1-GluA4) with GluA1/GluA2 (comprising ~80% of all synaptic AMPARs) and GluA2/GluA3 heteromers being the predominant conformation (Wenthold et al., 1996; Lu et al., 2009), whereas developmentally regulated GluA4 is mostly absent in mature excitatory neurons (Zhu et al., 2000). Each AMPAR subunit exhibits similar core structure with a variable cytosolic c-tail which enables protein-protein interactions and post-translational modifications (reviewed in Henley et al., 2011; Huganir and Nicoll, 2013). The c-tail of the different GluA subunits has been postulated to be a critical factor in AMPAR trafficking. The long c-tail of the GluA1 subunit has attracted the most attention because is a primary target of calcium/calmodulin-dependent protein kinase II (CaMKII), an important molecule for memory formation and LTP (Lisman and Goldring, 1988; Silva et al., 1992). CaMKII-mediated phosphorylation of the GluA1 c-tail stabilizes receptors at synapses through a PDZ-dependent mechanism which suggested that incorporation of GluA1-containing AMPARs into synapses is a major mechanism underlying LTP (Hayashi et al., 2000; Plant et al., 2006). Because GluA1 homomers are calcium permeable (Sans et al., 2003), in contrast to GluA1/GluA2 heterodimers, it has been proposed that a transient insertion of GluA1-containing AMPARs is an important step during LTP induction (Plant et al., 2006). These newly incorporated calcium permeable receptors could magnify the calcium influx at synapses resulting in LTP stabilization during the first minutes of potentiation. However, regular synapses contain extremely low levels of GluA1 homomers (Lu et al., 2009), thus it has been proposed that LTP maintenance is subsequently supported by the steady replacement of GluA1 by GluA2-containing receptors (Shi et al., 2001; Plant et al., 2006; Yang et al., 2010; Jaafari et al., 2012).

Consistent with this model, GluA2 and GluA3 subunits appear to be the primary targets during constitutive trafficking of AMPAR endocytosis during LTD. For example, constitutive trafficking of GluA2 is regulated by the multimeric ATPase N-ethylmaleimide sensitive factor (NSF) since blockade of the GluA2-NSF interaction results in a rapid run-down of AMPAR-mediated currents (Nishimune et al., 1998). In addition, the short c-tails of both GluA2 and GluA3 subunits display PDZ-interacting motifs which mediate the binding to several synaptic molecules. One of these motifs allows the binding to the protein interacting with C-kinase 1 (PICK1). PICK1-dependent interactions selectively regulate the constitutive and activity-dependent recycling of GluA2/GluA3-containing receptors by facilitating the formation of functional protein complexes that involve molecules like the memory-associated Kidney/BRAin protein KIBRA (Kim et al., 2001; Lin and Huganir, 2007; Citri et al., 2010; Makuch et al., 2011; but see also Terashima et al., 2008). Furthermore, another PDZ domain-containing protein, the glutamate receptor-interacting protein 1 (GRIP1), has also been implicated in specifically stabilize GluA2 and GluA3 subunits at synapses (Dong et al., 1997).

These findings have promoted a widely accepted model in which during LTP GluA2-lacking AMPARs are rapidly inserted at synapses likely by laterally diffusing from extrasynaptic localizations. Both synaptic and extrasynaptic AMPARs can be rapidly replenished by regulated exocytotic events providing enough receptors to engage in both activity-dependent and constitutive trafficking (Passafaro et al., 2001; Makino and Malinow, 2009; Jurado et al., 2013; Arendt et al., 2015). Subsequently, GluA2-lacking AMPARs can be steadily replaced by GluA2-containing receptors which are more susceptible of dynamic regulation during baseline transmission and LTD (Shi et al., 2001; Plant et al., 2006; Yang et al., 2010; Jaafari et al., 2012; see model of AMPAR trafficking in Figure 1). However, this prevailing view has recently been challenged. Using a molecular replacement approach in which different combinations of GluA1 c-tail mutants replaced the endogenous subunit, Granger et al. (2013) showed that AMPAR subunit composition is not a definitive determinant for LTP. These findings also exposed that the insertion of different glutamate receptors such as kainate receptors can support synaptic potentiation. These results shed new light into the mechanisms of synaptic plasticity and imply that the most important requirement for LTP is the rapid recruitment of glutamate receptors at synaptic localizations independently of subunit composition. Furthermore, using organotypic slices Watson et al. (2017) have recently shown that the AMPAR N-terminal domain may be required for LTP by mediating synaptic anchoring in a subunit-selective manner. Mutagenesis experiments revealed that AMPARs lacking the N-terminal domain are more labile and unable to sustain LTP while synaptic depression was enhanced suggesting that AMPAR anchoring through the N-terminal domain is important for maintaining normal synaptic strength and LTP expression. These recent advances prompt new interesting questions on AMPAR dynamics and regulation and will produce exciting avenues of investigation in the near future.

**Figure 1:** α-amino-3-hydroxy-5-methyl-4-isoxazolepropionic acid receptor (AMPAR) trafficking in healthy and aged brain. Top panel: AMPAR trafficking in the healthy brain. Central panel: *AMPAR trafficking during basal transmission*: AMPARs heterodimers are stabilized at the PSD through an indirect interaction with PSD-95 mediated by stargazin. Synaptic GluA3/GluA2 heterodimers are highly dynamic and undergo constitutive recycling via recycling endosomes. Phosphorylation levels of S845 of GluA1 c-tail are low perhaps by maintaining protein kinase A (PKA) and protein kinase C (PKC) away from synapses. These kinases bind to protein scaffold AKAP150 which may be recruited to synaptic compartments in response to neuronal activation. Left Panel: *AMPAR internalization during long-term depression (LTD)*: mild calcium influx through N-methyl-D-aspartate receptors (NMDARs) activates dephosphorylation of S845 in a calcineurin-dependent manner. Upon calcium influx AKAP150 is concentrated at the PSD where serves as a synaptic anchor for calcineurin. Calcineurin-dependent dephosphorylation destabilizes the interaction of AMPARs with the PSD thus promoting a lateral move to the dendritic shaft where receptors are later internalized by vesicular compartments. Simultaneously, calcium binding to protein interacting with c-kinase 1 (PICK1) elicits an open (active) conformation that accelerates the endocytosis of GluA3/GluA2 receptors. Other molecules involved in the PIP3 pathway such as PTEN are recruited to the PSD via a PSD-95-dependent mechanism. PTEN activation at synapses reduces the levels of PIP3 in the plasma membrane destabilizing AMPARs. Reduction of PIP3 may activate GSK3β which also facilitates AMPAR removal through an unidentified mechanism. Right Panel: *AMPAR insertion during long-term potentiation (LTP)*: high frequency stimulation induces a strong activation of NMDARs sufficient to recruit CaMKII to the synapse where it phosphorylates S381 of the GluA1 subunit thereby increasing channel conductance and synaptic stability. Other kinases like PKA and PKC may approach synaptic targets due to AKAP150 translocation to synapses thus increasing the phosphorylation levels of other critical residues such as S845. Calcium influx promotes postsynaptic exocytosis of AMPARs more likely at the dendritic shafts (schematics represent exocytosis within the dendritic spine for simplicity). Exocytosis of GluA1-containing receptors may occur during the first minutes but then are steadily replaced by GluA2-containing AMPARs. Recently inserted receptors laterally diffuse to the PSD where can are trapped by new synaptic slots which theoretically could accommodate different types of glutamate receptors. Bottom panel: AMPAR trafficking in the aged brain. Central panel: *AMPAR trafficking during basal transmission*: basal transmission is decreased as a consequence of healthy aging. Synaptic GluA3/GluA2-containing AMPARs are not replenished at the same rate than at younger synapses inducing weaker synaptic transmission. In addition phosphorylation levels may be altered. Disruptions in critical scaffolding molecules like PSD-95 may contribute to alterations of synaptic structure and morphology. Left Panel: *AMPAR internalization during LTD*: internalization of AMPARs in enhanced in older synapses likely as a consequence of an increased endocytosis rate and changes in phosphorylation levels. Right Panel: *AMPAR insertion during LTP*: LTP is impaired in older synapses where newly inserted AMPARs may be easily removed from an unstructured PSD undergoing enhanced endocytosis.

### AMPAR Phosphorylation

Phosphorylation is a critical determinant of AMPAR trafficking and function (recently reviewed in Lu and Roche, 2012; Wang et al., 2014). In general, kinase activity resulting in AMPAR phosphorylation is associated with LTP whereas phosphatase activity and dephosphorylation is linked to LTD (Lee et al., 2000). An important phosphorylation target for both CaMKII and protein kinase C (PKC) is the serine 831 (S831) in the long GluA1 c-tail which leads to an increase of channel conductance (Roche et al., 1996; Derkach et al., 1999; Kristensen et al., 2011). Work in transgenic mice expressing mutated versions of GluA1 CaMKII sites has revealed a potential role of this particular phosphorylation event during synaptic plasticity and memory retention (Lee et al., 2003, 2010, but see also Granger et al., 2013).

Phosphorylation of another GluA1 residue (S845) by protein kinase A (PKA) also increases the peak conductance and open probability of the channel (Banke et al., 2000). PKA-mediated phosphorylation of GluA1 S845 stabilizes extrasynaptic GluA1 homomers, to become more readily available to reach synapses during LTP whereas S845 dephosphorylation facilitates AMPAR endocytosis during LTD (He et al., 2009). GluA1 S845 is dephosphorylated by the calcium dependent phosphatase calcineurin (also known as PP2B). Interestingly, calcineurin and PKA can be jointly anchored by synaptic scaffold AKAP150 which brings together these two antagonistic functions at synapses. A specific AKAP150 knockdown or the expression of a mutant unable to bind calcineurin lead to enhanced GluA1 S845 phosphorylation and blocked LTD, but not LTP (Jurado et al., 2010b; Sanderson et al., 2012) consistent with the idea that the net balance of AMPAR phosphorylation determines receptors’ stability at synapses. Additionally, phosphatases and kinases involved in the PIP3 pathway have been shown to regulate AMPAR dynamics during LTP and LTD (Man et al., 2003; Arendt et al., 2010; Jurado et al., 2010a). However this form of regulation is likely to recruit several converging pathways rather than directly affect AMPAR phosphorylation.

Given the importance of AMPAR phosphorylation in regulating receptor activity, it has been proposed that phosphorylation levels are maintained low during baseline conditions and then regulated by neuronal activity (Hosokawa et al., 2015). This may explain why changes in AMPAR phosphorylation show more profound effects during activity-dependent than constitutive trafficking. Although further work is required to elucidate the exact mechanisms, the present evidence highlights an important role of phosphorylation, and surely other post-transcriptional modifications like palmitoylation and ubiquitylation (Lu and Roche, 2012), in controlling AMPAR trafficking and function. In this regard, ubiquitylation and phosphorylation may be strategic targets during neurodegenerative diseases as it has been shown that soluble Aβ oligomers increase AMPAR ubiquitination (Rodrigues et al., 2016) and reduce phosphorylation of GluA1 S845 occurring simultaneously to AMPAR removal from the plasma membrane (Guntupalli et al., 2017; Widagdo et al., 2017).

### Other Pathways of AMPAR Regulation

Protein-protein interactions play also a crucial role in AMPAR dynamics. AMPAR regulatory proteins such as the canonical transmembrane AMPAR regulatory proteins (TARPs) serve as auxiliary subunits that regulate channel activity and synaptic stabilization (Bats et al., 2007; Coombs and Cull-Candy, 2009). Although the TARP family is the best known, there has been a great progress in identifying novel AMPAR auxiliary subunits (recently reviewed in Jackson and Nicoll, 2011) along with adhesion molecules such as leucine-rich repeat transmembrane (LRRTM) proteins and N-cadherins (Saglietti et al., 2007; Soler-Llavina et al., 2013) which also contribute to synaptic retention.

TARPs such as stargazin and γ5 are key regulators of AMPAR biophysical properties by reducing the sensitivity to polyamines of GluA2-lacking receptors (Soto et al., 2007, 2009). In addition to these modulatory roles, TARPs participate in AMPAR trafficking and synaptic retention. For example, stargazin and TARPs γ3, γ4 and γ8 stabilize synaptic AMPARs through binding to PSD-95 and this stabilization has been postulated to be important during LTP (Tomita et al., 2005). During high frequency stimulation, glutamate binding to AMPARs reduces the interaction with stargazin which destabilizes desensitized receptors to diffuse away from synapses (Morimoto-Tomita et al., 2009; Constals et al., 2015; but see also Nakagawa et al., 2005). This mechanism may remove inactive AMPARs from synapses to be later replenished by fresh receptors from extrasynaptic compartments to sustain LTP. Although it has not fully been elucidated, there is accumulating evidence that some TARPs including stargazin may differentially affect AMPAR trafficking depending on subunit composition. For example in the absence of stargazin, there is an increase in GluA1-containing AMPARs in synapses suggesting that these receptors can reach synaptic compartments independently of this molecule (Bats et al., 2012; but see also Jackson et al., 2011). Future work will examine how AMPAR auxiliary subunits coordinate their multimodal roles to regulate channel activity, subunit composition and synaptic retention.

## AMPAR Signaling during Normal Aging

Before deepening into AD pathology, it is important to consider how the molecular processes that govern AMPAR-mediated transmission are affected during healthy aging. An older brain often exhibits mild defects in cognitive capabilities such as spatial and working memory with usually harmless consequences. This natural cognitive decline does not seem to be directly connected to significant neuronal loss which only seldom occurs in healthy elderly, but rather depends on the reorganization of synaptic structure (recently reviewed in Morrison and Baxter, 2012) suggesting abnormalities in the trafficking and stabilization of synaptic molecules.

To date, work focused in the events underlying healthy aging are limited to just a few studies tangentially addressing AMPAR trafficking by the means of analyzing synaptic plasticity. The primary findings of these studies conclude that in general LTP in older animals is less robust and requires stronger stimulation protocols to be elicited (Moore et al., 1993; Barnes et al., 2000; Tombaugh et al., 2002) whereas LTD appears to be facilitated (Norris et al., 1996). These findings suggest that the machinery involved in AMPAR removal from synapses may be enhanced later in life. This mechanism acting during natural aging may be exploited by Aβ or other pathological metabolites to further decrease synaptic AMPARs and trigger synaptic decline (Kamenetz et al., 2003; Hsieh et al., 2006; Shankar et al., 2007).

A surge of instability at the postsynaptic density may have negative repercussions not only for synaptic plasticity but also for maintaining stable synaptic strength. In fact, overall AMPAR hypofunction in aged subjects is suspected however it is uncertain whether this is a consequence of a decrease in synaptic AMPARs or an increase of modified receptors with reduced stability at synapses and/or conductivity. Two recent studies in aged rats showed that the administration of positive allosteric modulators of AMPARs had a beneficial effect on restoring age-related memory and synaptic potentiation deficits (Bloss et al., 2008; Radin et al., 2016). These results imply that at older synapses the number of functional AMPARs is sufficient to support LTP and memory storage but these receptors are mostly silent in the absence of appropriate enhancers.

The aforementioned scenario suggests two alternative hypotheses. One theory could postulate that aging alters presynaptic function thereby reducing glutamate release. A decrease in glutamate exocytosis would particularly affect AMPARs which bind to the endogenous agonist with much lower affinity than other glutamate receptors such as NMDARs (Edmonds et al., 1995). In fact, a significant increase in the bouton size and number of synaptophysin-positive terminals has been reported in the hippocampus of aged rats (Shimada et al., 2003; Himeda et al., 2005) suggesting that aging may hinder glutamate release leading to enlarging presynaptic compartments as a compensatory mechanism.

A second scenario could predict an increase of modified AMPARs which are either more labile at synapses or with reduced net conductivity. In this situation the administration of stimulants may overcome their loss of function, at least transiently. As discussed previously, increased instability and reduced conductivity can be triggered by altering AMPAR phosphorylation and/or by modifying their subunit composition. Currently, there are no reports assessing AMPAR phosphorylation in animal models of normal aging however a study by Hara et al. (2012) suggested that a switch in AMPAR subunit composition may be involved in natural cognitive decline. They used electron microscopy to analyze the subcellular localization of both the GluA2 subunit and protein kinase PKMζ in young and aged monkeys. Their results showed that older animals presented less synapses co-labeled with GluA2 and PKMζ. It is interesting that GluA2-containing AMPARs are targeted in other brain pathologies like epilepsy (Grooms et al., 2000) however it is unknown whether age related mechanisms specifically target these receptors or whether their exit from synapses is a consequence of a broader reorganization of synaptic architecture. Given that most AMPARs in mature cortical and hippocampal synapses are GluA1/2 heteromers (Lu et al., 2009), it is reasonable to propose that mechanisms directed to remove GluA2 will greatly affect synaptic transmission and plasticity in the aging brain (see model of AMPAR trafficking in healthy aging in Figure 1). Despite these recent advances, studies exploring AMPAR dynamics in neurons from naturally aged subjects are scarce thus it is still unclear whether AMPAR phosphorylation and/or subunit composition are differentially regulated in older brains and how these alterations may contribute to cognitive decay.

## AMPAR Signaling During Neurodegeneration: Focus on Alzheimer’S Disease

In the pathology of AD, neuronal function is compromised in two fronts: extracellularly by the accumulation of secreted Aβ oligomers and intracellularly by deposits of aberrant tau protein. However it is possible that neurons may not have to face these challenges simultaneously. Cellular and animal models indicate that Aβ accumulation precedes NFTs formation (Hardy and Selkoe, 2002) suggesting that both metabolites may take part in different stages during the progression of neurodegeneration. Here, I discuss some of the recent work analyzing the roles of Aβ and NFTs in AMPAR trafficking and how these molecules may work synergistically to alter synaptic structure and function.

### Effect of Aβ in AMPAR Signaling

#### Aβ in Synaptic Plasticity

Aβ induces synaptic aberrations by altering the morphology and composition of synapses that lead to significant dendritic spines loss (Lacor et al., 2007; Bittner et al., 2010). These effects suggest a critical role of Aβ in altering synaptic function. In fact, the most consistent effect in response to exogenous Aβ or APP overexpression is the induction or enhancement of synaptic depression by a process analogous to Hebbian LTD (Kamenetz et al., 2003; Hsieh et al., 2006; Shankar et al., 2007). Similarly to canonical LTD, Aβ-induced depression requires NMDARs activation which triggers the removal of AMPARs from synapses (Kamenetz et al., 2003; Hsieh et al., 2006; Shankar et al., 2007). Furthermore, the blockade of AMPAR endocytosis prevents the loss of dendritic spines induced by Aβ (Hsieh et al., 2006). Interestingly, Aβ oligomers have been proposed to indirectly interact with NMDARs (Decker et al., 2010) which may lead to neuronal oxidative stress (De Felice et al., 2007). According to the requirement of NMDAR activation, the removal of synaptic AMPAR in response to Aβ has been proposed to share common signaling pathways with LTD. For example, blocking LTD-related pathways like p38 MAPK and calcineurin prevented Aβ-induced LTP deficits and AMPAR internalization (Wang et al., 2004; Zhao et al., 2010). Additionally, the inhibition of GSK3β and PTEN, two molecules involved in the PIP3 pathway which have been involved in activity-dependent regulation of dendritic growth and LTD (Arendt et al., 2010; Jurado et al., 2010a; Rui et al., 2013), restored Aβ-induced AMPAR endocytosis (Rui et al., 2010) and protected synaptic function and cognition in cellular and animal models of AD (Knafo et al., 2016). Despite these similarities, Aβ-induced synaptic depression has also been proposed to engage distinct signaling cascades such as the metabotropic function of NMDARs by targeting GluN2B-containing receptors which recruit protein G-dependent pathways (Kessels et al., 2013).

In accordance with synaptic and cognition decline, LTP is impaired in animal models of AD and in response to acute administration of Aβ (Walsh et al., 2002; Shankar et al., 2008; Wei et al., 2010). One of the main effects of Aβ is to alter CaMKII synaptic localization. Using cortical neurons from APP transgenic mice, Gu et al. (2009) found that he synaptic pool of CaMKII was significantly reduced in an APP transgenic mouse. This effect was consistent with a decrease in the density of CaMKII clusters at synapses of cortical neurons treated with Aβ oligomers (Gu et al., 2009). Conversely, overexpression of CaMKII restored AMPAR-mediated transmission suggesting that Aβ alters the subcellular distribution of CaMKII which in turn destabilizes synaptic AMPARs and hinders synaptic potentiation. Alternatively, soluble Aβ may affect LTP induction by reducing surface expression of NMDARs (Snyder et al., 2005). However, a decrease in surface NMDARs may in turn have a protective effect since a specific NMDAR knock-down abolished the binding of oligomers to dendrites suggesting that NMDARs might be required for the synaptic targeting of Aβ (Decker et al., 2010). Furthermore, Aβ has been proposed to specifically activate GluN2B-containing NMDARs leading to neuronal hyperactivation and LTP blockade (Li et al., 2009, 2011). Another route that Aβ may utilize to interfere with AMPAR insertion appears to be interfering with BDNF-dependent pathways required for synaptic potentiation (Garzon et al., 2002; Peng et al., 2009). This accumulative evidence indicates that soluble Aβ oligomers underlie synaptic dysfunction by altering both NMDARs and AMPAR trafficking and function (reviewed in Tu et al., 2014).

#### Synaptic Targets of Aβ: A Role for AMPARs Subunits?

Intriguingly, the presence of Aβ plaques do not necessarily lead to neurodegeneration (Mintun et al., 2006; Quigley et al., 2011; Wirth et al., 2013) posing the question of why certain people retain their cognitive function while others develop dementia. A potential explanation could be that Aβ-induced toxicity requires the activation of additional factors which expression may be highly variable in the population. But, what are these additional factors or binding partners of extracellular Aβ? To date the most widely accepted partner of Aβ is the cellular prion protein (Laurén et al., 2009) which has led to hypothesize that Aβ itself could behave as a self-propagating prion to induce neurodegeneration (Watts and Prusiner, 2017). More recently, a pull-down approach has been used to identify endogenous binding partners of Aβ oligomers from cerebrospinal fluid (Rahman et al., 2015). Approximately 100 molecules primarily involved in lipid metabolism, homeostasis and the immune response have been identified (Rahman et al., 2015) suggesting that Aβ may affect multiple cellular functions through a myriad of potential binding partners.

Interestingly, Aβ oligomers have been shown to preferentially target different AMPAR subunits (Zhao et al., 2010; Reinders et al., 2016). Using co-immunoprecipitation and photoreactive amino acid cross-linking in primary hippocampal cultures, Zhao et al. (2010) showed that Aβ oligomers preferentially affect GluA2-containing AMPARs raising the possibility that Aβ may alter AMPAR trafficking by binding directly to the GluA2 protein complex. Additionally, GluA2-containing AMPARs appear to be primarily affected during healthy aging (Hara et al., 2012) suggesting that Aβ signaling may exploit a naturally occurring mechanism to aggravate ongoing synaptic decay. However, a recent study suggested that another AMPAR subunit may be Aβ preferred target. Reinders et al. (2016) showed that synaptic depression and spine loss in CA1 neurons that overexpressed Aβ required GluA3 expression. In their electrophysiology experiments, LTP remained unaltered in acute hippocampal slices from GluA3-deficient mice in response to exogenous Aβ which efficiently diminished LTP in control mice. These results imply that Aβ preferentially drives GluA3-containing AMPAR removal. This apparent contradiction may be explained when considering that most GluA3 heteromers exist as GluA2/GluA3-containing AMPARs (Lu et al., 2009). A model then arises in which Aβ oligomers favorably bind GluA2/GluA3-containing AMPARs thereby triggering the selective endocytosis of these receptors from the surface of synapses (see model of how Aβ alters AMPAR trafficking in Figure 2). A potential target for Aβ to jointly alter GluA2/3-containing AMPAR recycling is PICK1 (Kim et al., 2001; Lin and Huganir, 2007; Citri et al., 2010). PICK1-dependent internalization is mediated by the phosphorylation of the GluA2 or GluA3 c-tails by PKCα, a process that leaves surface GluA1-containing receptors mostly unchanged (Kim et al., 2001; Lin and Huganir, 2007; Citri et al., 2010; but see also Terashima et al., 2008). Remarkably, synapses from mice lacking PICK1 are protected from Aβ-induced depressive effects (Alfonso et al., 2014) indicating that interaction of PICK1 with GluA2/3 AMPARs may play a role in Aβ synaptotoxicity.

**Figure 2:** Effect of soluble amyloid-β (Aβ) oligomers and hyperphosphorylated tau in AMPAR trafficking. Top panel: effect of soluble Aβ oligomers in AMPAR trafficking: Central panel: *AMPAR trafficking during basal transmission*: soluble Aβ oligomers may bind to NMDARs and AMPARs (preferentially to GluN2B and GluA2/GluA3 heteromers). This interaction enhances AMPAR endocytosis which decreases synaptic strength. Left Panel: *AMPAR internalization during LTD*: in the presence of Aβ, NMDAR-dependent LTD engages similar signaling pathways than regular LTD. However, endocytosis exacerbation may contribute to increase synaptic depression through a PICK1-dependent mechanism. Right panel: *AMPAR insertion during LTP*: accumulation of Aβ oligomers prevents CaMKII from reaching synaptic localizations and blocking AMPAR phosphorylation important for LTP expression. Bottom panel: effect of hyperphosphorylated tau in AMPAR trafficking. Central panel: *AMPAR trafficking during basal transmission*: hyperphosphorylated tau is missorted to dendritic spines where dysregulates key components of the PSD such as PSD95 and NMDARs. Hyperphosphorylated tau prevents Fyn kinase from reaching synaptic localizations which may alter basaline phosphorylation levels of both AMPARs and NMDARs. Left Panel: *AMPAR internalization during LTD*: as a consequence of reduced PSD stability, LTD may appear enhanced in the presence of hyperphosphorylated tau at synapses. Right Panel: *AMPAR insertion during LTP*: insertion of AMPARs may not be affected by hyperphophorylated tau, however subsequent synaptic retention may be impaired due to a less stable PSD. Additionally, the inability of critical protein kinases such as the Fyn kinase to reach their synaptic target may contribute to a loss of newly-inserted receptors.

#### Targeting AMPAR Subunits: A Novel Therapeutic Approach for AD?

By inducing the selective endocytosis of GluA2/3s, Aβ could trigger synaptic depression and reduce synapse stability. Thus it seems reasonable to speculate that synapses which reduced levels of GluA2/3-containing AMPARs may be protected from Aβ toxicity. In fact, a recent screening for gene-expression profiles associated with mild cognitive impairment found GluA3 among the genes that showed a strong negative correlation with neurodegeneration (Berchtold et al., 2014). Synapses with lower levels of GluA2/3 may be generated during synaptic potentiation since it has been proposed that GluA1-containing AMPARs are primarily inserted during LTP (Hayashi et al., 2000; Plant et al., 2006; but also see Granger et al., 2013). However future therapeutic approaches based on reducing GluA2/3 AMPARs in favor of GluA1 could have unexpected side effects. Although in general soluble Aβ facilitates synaptic depression and hinders potentiation, intracellular Aβ has also been shown in some cases to increase GluA1-containing AMPARs which in turn may lead to calcium-dependent excitotoxicity (Whitcomb et al., 2015). Despite pharmacological approaches targeted to potentiate synaptic strength by recruiting GluA1-containing AMPARs may present some undesirable side effects, it seems reasonable to postulate that maintaining an intellectually active life style may protect from some of the molecular alterations triggered by Aβ plaques which normally appear in naturally aging brains (Mintun et al., 2006; Quigley et al., 2011; Wirth et al., 2013).

### Effect of NFT in AMPAR Signaling

#### Effect of NFT in Synaptic Transmission

Although the role of tau in disrupting AMPAR trafficking has been less studied than the effect of oligomeric Aβ, there is substantial evidence of synaptic abnormalities associated with tau-mediated signaling with numerous studies exposing that AMPARs appear particularly vulnerable to tau pathology. These body of work described a significant loss of surface receptors in cultured neurons treated with mutated tau proteins (Hoover et al., 2010; Yu et al., 2012) and in tau mutant mice (Eckermann et al., 2007; Yoshiyama et al., 2007; Mocanu et al., 2008; Polydoro et al., 2009; Bittner et al., 2010; Rocher et al., 2010; Crimins et al., 2011; Sydow et al., 2011) with a few studies reporting no changes in synaptic density or morphology (Shahani et al., 2006; Tackenberg and Brandt, 2009; Kimura et al., 2010; Rocher et al., 2010). Reconciling these contradictory results is complicated by the multiple tau manipulations employed ranging from human mutant and wild type isoforms, pro- or non-aggregated, fluorescent-tagged and endogenous tau in *in vitro* and* in vivo* models. To complicate things further, in recent years there has been a growing appreciation that NFTs may be less efficient in disrupting neuronal function than soluble tau (de Calignon et al., 2009; Spires-Jones et al., 2009; Fox et al., 2011), thus tau pathology and synaptotoxicity may greatly depend on the ratio between the aggregated and dissociated forms. However reorganization of synaptic ultrastructure may occur without a dramatic remodeling of the synaptic density. A recent report addressed the effect of tau on synapses using novel array tomography and two-photon *in vivo* microscopy in an animal model of taupathy (rTg4510; Santacruz et al., 2005; Kopeikina et al., 2013). These results revealed that although synaptic density remained unaltered critical synaptic proteins including PSD-95, GluN1 and GluA1 were reduced. These findings suggest synapses exposed to aberrant tau may exhibit subtle changes at the ultrastructural level which in the long-run may significantly affect synaptic function.

#### Effect of NFTs in Synaptic Plasticity

As aforementioned, there is ample evidence indicating that synaptic strength is altered in models of tau abnormalities (D’Amelio et al., 2011; but see also Crimins et al., 2011) and that synaptic plasticity appears disrupted as a consequence of aberrant tau. Polydoro et al. (2009) exposed that basal synaptic transmission and induction of LTP with high-frequency stimulation is perturbed in hippocampal CA1 region of old but not young htau transgenic mice reinforcing the notion that tau-dependent signaling interferes with AMPAR trafficking and synaptic plasticity later in life (Kremer et al., 2011). Interestingly, recombinant human tau oligomers have been shown to block LTP and induce memory impairments independently of Aβ (Fá et al., 2016). However another study detected no effect in LTP but rather an enhancement of LTD (D’Amelio et al., 2011). These discrepancies may be a consequence of employing two different transgenic models. While Polydoro et al. (2009) used the htau mice which overexpress human tau (Andorfer et al., 2003), D’Amelio et al. (2011) employed Tg2576, a common model of AD that overexpresses human Aβ (Hsiao et al., 1996). Given that Aβ facilitates LTD, it may be plausible that increased Aβ levels in Tg2576 mice could conceal tau-dependent effects in synaptic potentiation. Despite these differences, there is a growing body of evidence indicating a crucial role of tau-dependent signaling in regulating synapse structure and function.

### Mechanisms of NFT-mediated Synaptotoxicity

But how a microtubule-associated protein, mostly located at presynaptic compartments may affect postsynaptic organization and dynamics? A potential explanation may lay in recent findings showing that tau can be localized not only in axonal microtubules but also at postsynaptic densities, albeit at much lower levels (Ittner et al., 2010). Particularly, hyperphosphorylated tau, but not a phosphorylation-deficient tau, is accumulated in dendritic spines where can dysregulate AMPAR trafficking together with key signaling molecules (Hoover et al., 2010; Zempel et al., 2010). Synaptic impairments originated by tau missorting seem to occur independently of neurodegeneration (Hoover et al., 2010) suggesting that tau may contribute to synaptic malfunction before evident cognitive deficits arise. In addition to interrupting AMPAR trafficking, tau can have disruptive effects in crucial signaling pathways. For example, postsynaptic tau has been shown to assist during the translocation of the Src kinase Fyn to dendritic spines (Ittner et al., 2010). Fyn kinase is a key regulator of GluN2 subunits phosphorylation which contributes to the stabilization of synaptic NMDARs through a PSD-95-dependent mechanism (Tezuka et al., 1999). Missorted tau to synapses disrupts postsynaptic targeting of Fyn kinase with negative effects in synaptic function and cognition (Bhaskar et al., 2005; Ittner et al., 2010), and conversely its deletion reduced the severity of spontaneous and chemically induced seizures in mice overexpressing Fyn (Roberson et al., 2011).

Although phosphorylated tau is usually considered potentially neurotoxic, recent evidence suggests a critical role of phosphorylated tau in maintaining normal synaptic transmission and plasticity. Thereby, using biochemical and electrophysiological assays, Regan et al. (2015), have shown that site-specific phosphorylation at serine 396 of tau is required for hippocampal LTD. Moreover, a recent report from Ittner et al. (2016) exposed positive effects of early tau phosphorylation in an animal model of AD. Particularly, mimicking tau phosphorylation at threonine 205 alleviated Aβ-induced neuronal death and offered protection from excitotoxicity during early stages of the disease (Ittner et al., 2016). These data challenge the idea that tau phosphorylation may be a negative consequence of Aβ synthesis and accumulation. Furthermore, tau-mediated mechanisms may be recruited as potential compensatory mechanisms during early AD prompting the intriguing possibility that activating tau phosphorylation during the initial phases of neurodegeneration may be beneficial. These findings certainly warrant future studies to determine how tau may be involved in inducing cognitive impairments by affecting synaptic function (see model of how tau alters AMPAR trafficking in Figure 2).

In addition to phosphorylation, tau acetylation is emerging as an interesting target of tau regulation during pathological aging as abnormal acetylation of tau lysines K274 and K281 have been associated with dementia in AD (Tracy et al., 2016; Tracy and Gan, 2017). Transgenic mice expressing human tau with lysine-to-glutamine mutations exhibit AD-related memory deficits and impaired hippocampal LTP. Interestingly, enhanced tau acetylation disrupts hippocampal synaptic plasticity, reduces postsynaptic KIBRA and is associated with loss of KIBRA expression in AD patients with dementia (Tracy et al., 2016; Tracy and Gan, 2017). Taken together these results suggest that strategies targeted to block tau acetylation may lead to effective treatments for cognitive decline in AD.

### Aβ and Tau Converging Pathways

Aggregates of Aβ oligomers and NFTs are hallmarks of AD, however it remains unknown how extracellular Aβ and intracellular NFTs trigger synaptic dysfunction. Do they employ different mechanisms or share common pathways to accelerate synaptic decline? There are also questions regarding the time-course of AD progression. Since pathological effects associated with plaques usually appear earlier (Hardy and Selkoe, 2002), it has been proposed that Aβ initiates synaptic alterations which are later exacerbated by NFTs. However the existence of tauophaties and the ability of hyperphoshorylated tau in altering synaptic transmission in the absence of neurodegenerative symptoms (Hoover et al., 2010) suggests that tau may act in the absence of Aβ.

Despite the answer to these questions remains largely unknown, there is ample evidence of a causal association between oligomeric Aβ and tau (Rapoport et al., 2002; Roberson et al., 2007; Ittner et al., 2010; Shipton et al., 2011; Nussbaum et al., 2012; but see also Tackenberg and Brandt, 2009). Several studies have shown that tau deletion can protect from Aβ-induced synaptic loss and cognitive impairment in several animal models of AD (Roberson et al., 2007, 2011; Ittner et al., 2010; Vossel et al., 2010). One of the most plausible mechanisms linking the actions of Aβ and tau in pathology may involve the stimulation of tau phosphorylation through a signaling pathway initiated by Aβ. Hyperphosphorylated tau is missorted to postsynaptic densities where it may contribute to the synaptotoxic role of oligomeric Aβ (Zempel et al., 2010; Ittner and Götz, 2011). Consistent with this, Aβ oligomers isolated from brains of AD patients were sufficient to elicit tau hyperphosphorylation in cultured hippocampal neurons (Jin et al., 2011) and anti-Aβ antibodies protected from tau hyperphophorylation and neuritic degeneration (Jin et al., 2011). A potential point of converge for Aβ and tau at synapses may be NMDARs activation since their blockade has been shown to abolish both Aβ-induced dendritic spine loss and tau-dependent toxicity (Shankar et al., 2007; but see also Tackenberg and Brandt, 2009). Interestingly, it has been recently proposed that Aβ could control tau phosphorylation by stimulating glutamate release from astrocytes which activates extrasynaptic NMDARs (Talantova et al., 2013). These data agree with a model where Aβ-mediated signaling promotes tau phosphorylation which may lead to anomalous hyperphosphorylation and pathology (but see also Ittner et al., 2016). However, new findings using human pluripotent stem cell derived neurons from AD patients has exposed that increased tau phosphorylation at Thr231 depends on β-secretase activity (Israel et al., 2012) raising the possibility that Aβ-induced tau phosphorylation can engage an alternative pathway independent of Aβ signaling.

Regulation of tau by Aβ-mediated NMDARs activation entails that common signaling pathways linked to these receptors may be implicated in facilitating the pathological effects of both molecules. In agreement, GSK3β regulates both tau phosphorylation and Aβ production and its inhibition prevents Aβ-induced impairment of LTP and improve AD pathology (Shipton et al., 2011). In addition to sharing common signaling pathways it may be possible that as a result of increasing production of Aβ oligomers and NFTs at late stages of neurodegeneration both molecules could be found in enough amounts to directly interact with each other. This possibility is supported by a recent study using co-immunoprecipitation and immunohistology techniques. Using this approach Manczak and Reddy (2013) have exposed a potential interaction between Aβ oligomers and phosphorylated tau in both human and animal AD brains which increased with disease progression. It is thus possible that pathological interactions between oligomeric Aβ and NFTs are important intermediate steps during later stages of AD. Considering the current findings we could imagine a scenario in which Aβ and tau may converge at synapses by hijacking key synaptic pathways such as NMDAR-mediated transmission. These early events may exacerbate synaptic degeneration until a complete convergence of tau and Aβ signaling pathways, facilitated by direct interaction between the two at later stages (see model AMPAR trafficking in AD in Figure 3). Future in-depth studies will be necessary to determine the interplay of tau and Aβ in disrupting AMPAR dynamics and neurodegeneration.

**Figure 3:** AMPAR trafficking during Alzheimer’s disease (AD): early and later phases. **(A)** *AMPAR trafficking during early phase of neurodegeneration*: at early stages soluble Aβ oligomers may activate a NMDAR-dependent pathway that results in increased tau phosphorylation levels and further Aβ synthesis. A plausible candidate to mediate these effects is GSK3β which reduces synaptic transmission and enhances LTD. **(B)** *AMPAR trafficking during later phases of neurodegeneration*: combined effects of Aβ and hyperphosphorylated tau prevent LTP expression in altered synapses likely by preventing the action of key protein kinases such as CaMKII and Fyn kinase. Aβ and hyperphosphorylated tau could form synaptotoxic aggregates at the PSD that further aggravate synaptic decay.

## Concluding Remarks

The dynamic regulation of AMPARs is a crucial factor in supporting baseline synaptic transmission and plasticity. Thus AMPAR dysregulation underlies synaptic decay during natural and pathological aging. Over the last years, great progress has been made in understanding how AMPAR signaling is affected during neurodegenerative diseases such as AD in which both NFTs and Aβ disrupt glutamate receptors and their downstream pathways. Interestingly, several findings indicate that selective dysregulation of GluA2/3-containing AMPARs may be an important target during both natural and pathological aging. Removal of GluA2 has profound consequences in trafficking and AMPAR calcium permeability resulting in an increase of calcium influx which may contribute to neuronal excitotoxicity. Selective targeting of GluA3 and GluA2-containing AMPARs during pathological conditions suggests the intriguing possibility that the molecular mechanisms involved in their regulation may be the foundation of novel therapies for neurodegenerative diseases. In this regard, personalized medicine catered to various genetic backgrounds may be helpful to identify the potential underlying causes of synaptic malfunction in a case-by-case basis. In order to accomplish this, a better understanding of the molecular underpinnings involved in AMPAR trafficking in healthy synapses will be crucial.

## Author Contributions

SJ prepared the figures, wrote and edited the manuscript.

## Conflict of Interest Statement

The author declares that the research was conducted in the absence of any commercial or financial relationships that could be construed as a potential conflict of interest.

## Footnotes

^1^http://www.alz.org/facts/
